RETRACTED

# Effect of section thickness on microstructure and mechanical properties of compacted graphite iron for diesel engine applications

**DOI:** 10.1016/j.heliyon.2021.e05930

**Published:** 2021-01-29

**Authors:** Mahmoud A. Essam, Ahmed Y. Shash, Hassan Megahed, Emad El-Kashif

**Affiliations:** a Mechanical Engineering Dept., Higher Technological Institute (H.T.I), 10th of Ramadan City, Egypt; b Faculty of Engineering and Materials Science, German University in Cairo, Cairo, Egypt; c Mechanical Design and Production Dept., Faculty of Engineering, Cairo University, Cairo, Egypt

**Keywords:** Compacted graphite iron, Wall thickness, Vermicular microstructures, Mechanical properties

## Abstract

Compacted (vermicular) graphite iron (CGI) is used in many substantial applications because its vermicular microstructure has superior mechanical properties at higher temperatures. Production of vermicular graphite cast iron diesel engine cylinder block with various sections’ thicknesses is a great challenge especially, if compacted graphite iron is made by controlling the pouring duration. Investigations on microstructure and hardness have been conducted on four different thicknesses (5, 10, 15, and 20 mm) of compacted graphite iron. Results demonstrated that pouring duration affects both cooling rate, and Mg/S content. These two parameters to decide the nodularity percentage and the matrix microstructure. Longer pouring duration lowers Mg/S content and decreases the cooling rate for the similar section thickness, however shorter pouring duration acts in the opposite direction. Microstructure and hardness are also affected by casting sections with the same pouring duration through different cooling rates. An increase in the cross-sectional thickness for the same pouring duration decreases the rate of cooling that encourages the formation of compacted graphite with pearlitic rather than martensitic a matrix in addition to lowers the nodular graphite count. Magnesium fading and compacted graphite ratio increased with longer pouring duration. Hardness decreased with larger section thickness and longer pouring duration due to the elimination of the martensite phase in the matrix.

## 1 Introduction

Casting is a basic production technique particularly sand casting that is the most accommodating production method for large-size products. Owing to compacted graphite cast iron toughness, damping capacity, and thermal fatigue durability properties, it is involved in numerous applications like internal-combustion engine blocks, brake drums, and cylinder heads in trucks, vans, and Lorries [1, 2].

Compacted graphite cast iron composed of an iron matrix that consists of one or mixture of iron phases (pearlite, ferrite, austenite, etc.) and graphite of worm shape. Factors controlling compacted cast iron microstructure include alloying elements content, cooling rate, and therefore, the supplement heat treatment after solidification [3]. The cooling rate plays a huge effect on pearlite and graphite content ratios similarly because of the morphology of graphite formed hence the properties of the material [4, 5, 6].

RETRACTED

Graphite in compacted graphite cast iron appears in an exceedingly worm-like form with curved ends while etched surface appears coral like that decreased stress concentration levels compared with gray (flakes) cast iron. This morphology of graphite ends up to higher cohesion in material and resistivity of crack propagation subsequently shock absorbing and toughness [7]. This morphology has great stability at an elevated temperature that persuades compacted cast iron of high shock applications at high temperatures [8]. During a comparison to lamellar graphite cast iron using compacted graphite cast iron can reduce a load of cylinder block by 25% as compacted cast iron has higher fatigue limits [9].

The ASTM A842-85 standards specify that compacted cast iron has 80% of its graphite in worm shape, and increasing this ratio results in decreasing strength. The Cooling rate also affects the direction of compacted growth that consequently affects the thermal conductivity of the material [10]. As pearlite % increases the strength of compacted graphite cast iron increase [11, 12]. The Cooling rate also affects the direction of compacted growth that consequently affects the microstructure of the produced cast iron. The increasing cooling rate of compacted cast iron increases the coincidental of graphite to form nodules that decrease ductility and damping capacity [13, 14].

The rate of cooling depends on the casting section thickness and thermal conductivity of the mould material where the massive casting section incorporates a lower cooling rate. Diversity in section thickness in casting affects the microstructure together with the casting that hence affects the product strength [15, 16, 17, 18]. In previous work [14], the authors studied the effect of heat treatment and holding time or pouring duration on the identical compacted graphite iron. However, internal-combustion engine blocks are employed in the as-cast condition. Therefore, the as-cast microstructures should be investigated. The aim of the current work is to check the effect of cooling rate on vermicular graphite cast iron through solidification of various casting section thickness with two different pouring duration (10.5 and 17.5 min respectively).

## 2 Experimental procedure

### 2.1 Production of CGI

A moderate frequency induction furnace was used to produce compacted graphite cast iron that works at approximately 500–5000 Hz frequency current. The furnace charged with 6000 kg approximately. The used spheroidal pig iron is (GGG70) with the chemical composition in Table 1. The furnace temperature was maintained at 1600 °C approximately to melt CGI. An induction furnace was used to melt CGI manufacturing from tube of copper and a magnetic field with high frequency that created by current that passes through this coil that is cooled by using water.

RETRACTED

**Table 1:** Chemical composition of pig iron GGG70.

Chemical Composition %									
GGG 70	C	Si	Mn	P	S	Mg	Cu	Sn	Fe
	3.70	1.90	0.40	0.03	0.02	0.045	0.03	0.06	Balance

The compacted graphite iron (CGI) was produced using step block casting in green sand with four different thicknesses 5, 10, 15 and 20 mm thick steps where the direction of tensile test samples are shown in Figure 1 with the chemical composition is shown in Table 2.

**Figure 1:** Step block cast with different thicknesses in mm.

**Table 2:** Chemical composition of compacted graphite iron.

Chemical Composition %											
Sample #	C	Si	Mn	P	S	Mg	Cu	Sn	Ti	Fe	Pouring Time (min.)
Sample 1	3.65	2.55	0.24	0.045	0.019	0.031	1.00	0.05	0.0091	Balance	10.53
Sample 2	3.65	2.51	0.24	0.046	0.015	0.021	0.98	0.05	0.0085	Balance	17.53

The charge was around 750 kg, the additives to transfer GGG70 to CGI were: 1) 1.5 kg ferrotitanium alloy with 80% Ti, 2) 0.5 kg pure tin (Sn) free of lead to enhance the mechanical properties and 3) 1% pure copper (Cu).

Compacted graphite cast iron was produced by the ladle treatment method. This method is one in all the foremost important techniques with **relevance** adding alloying elements to the molten iron throughout production. Steel scrap, spheroidal graphite (SG iron), and ferrosilicon (FeSi) alloy were charged within the induction furnace to organize the desired CGI. The ladle of cast iron alloy should be maintained under adequate hydrostatic pressure of coming liquid of cast iron alloy. The charge of the ladle holds until magnesium fading complete. The ratio of magnesium fading is influenced by holding time, transport time, and pouring time. The treatment temperature varied within the range of 1430 °C–1480 °C, the two samples were poured at the various pouring time, and the primary pouring time for the first sample was 10.53 min, however, the second sample was 17.53 min.

### 2.2 Microstructure analysis and Brinell hardness

Optical microscopy was used to observe the microstructure of compacted graphite cast iron step blocks. The tested samples were prepared according to standard metallographic procedures. Step block with different thicknesses started from 5 mm to 20 mm stepped by 5 mm were taken from casted step block and mounted in bakalite, finally subsequent by grounding and polishing. Subsequently, the samples were etched by using a Nital solution of concentration 2%. This technique is chosen due to its consistency and uniformity. The photograph of the CGI samples was taken by optical microscope (A Zesiss Axiotech). Throughout this analysis; image analysis program and optical metallography were used to determine the percentage values of carbides, pearlite and martensite. The hardness was determined using the Brinell hardness test at a load of 1000 kg at the core of the specimens.

RETRACTED

### 2.3 Tensile test

Tensile test samples were produced according to standard ASTM E8M; these samples were taken from step bloc as shown in Figure 1. For each thickness, three repetition tensile specimens were machined for testing. A universal testing machine Walter + bai ag LFM-L 20KN were used to measure tensile strength at temperature approximately equal 25 °C. Each value of tensile properties represents the mean value for three tested samples.

## 3 Results & discussions

### 3.1 Effect of wall thickness on microstructure

One of the supreme essential properties in the microstructure of CGI is pearlite to ferrite matrix contents, so pearlite stabilizer elements for example copper and tin were used to enhance pearlite contents. The rate of cooling also affects the content on the pearlite matrix, so engine blocks that have higher carbon equivalent may have around 10% pearlite microstructure. The affinity of ferrite matrix to form in microstructure is high without using pearlite stabilizer elements, for example, Cu and Sn as stated formerly. The adding of these elements enhances the mechanical properties of CGI.

In this study to enhance a pearlite matrix in CGI, the Cu and Sn were added by 1 % and 0.045 respectively to accomplish approximately 80% pearlite matrix. A Measure of included copper and tin depends on the geometry of the item [11, 12]. The addition of these alloying elements shifts the C-curve to the right-hand side and promotes the formation of hard phases like martensite and pearlite rather than ferrite [19].

The casting of vermicular graphite cast iron product could be an inflexible issue when spheroidal (ductile), and flake (gray) graphite iron casting is taken into account because the formation of worm-shaped graphite particles is stable for a few restricted conditions. Moreover, provision of engine cylinder blocks face some difficulties that may be an interrelation between chemical composition of the alloy, cooling conditions, and physical characteristics like that complicity of geometric shape, volume and weight of casting that needs to suitable tolerance. Therefore, the casting chemical composition is to be composed with very sensibly to an adequate Mg level and requirement of inoculation. Actually, the chemical composition that can be used to synthesis of vermicular graphite cast iron in one foundry may be not suitable for another foundry [19]. Formations of CGI rely on magnesium ratio in addition to the Magnesium/Sulphur ratio. As shown in Table 3, to obtain a vermicular graphite cast iron can be achieved by setting two values, one of them is magnesium to sulphur ratio that may be around 1.5% and another value is the ratio of carbon equivalent that have a range between 4.40% to 4.50%. The following Figures 2 and 3 reveal the different thicknesses of microstructure of CGI before etching to show the nodularity percentage.

RETRACTED

**Table 3:** Spheroidal number and Brinell hardness values of specimens at different thicknesses.

Specimens	Section Thicknesses (mm)	Spheroidal No.	Brinell Hardness	Nodularity %	Carbon Equivalent	Mg/S ratio
Sample no. 1	5	150	315	32.65	4.50	1.63
	10	102	312	21.47		
	15	87	259	16.34		
	20	58	250	14.21		
Sample no. 2	5	106	250	23.10	4.48	1.40
	10	92	250	20.35		
	15	63	248	17.78		
	20	44	237	13.65

**Figure 2:** Nodularity % for sample number 1 with different thicknesses before etching: A) Wall thickness 5mm, nodularity % 32.65, B) Wall thickness 10mm, nodularity % 21.47,C) Wall thickness 15mm, nodularity % 16.34, and D) Wall thickness 20mm, nodularity % 14.21.

**Figure 3:** Nodularity % for sample number 2 with different thicknesses before etching: A) Wall thickness 5mm, nodularity % 23.10, B) Wall thickness 10mm, nodularity % 20.35,C) Wall thickness 15mm, nodularity % 17.78, and D) Wall thickness 20mm, nodularity % 13.65.

The technique for determining nodularity percentage for CGI is as follows:

• A microscopic image was captured before etching to investigate nodularity percent and a number of nodules.
• The graphite area was determined.
• Nodularity percentage = $\frac{\text{nodules count average value}}{\text{graphite area average value}}$
• The average of three measurements was taken for the number of nodules count and graphite area for each sample.

It was noticed that from a microstructure in Figures 2 and 3 shown above, the pouring time and wall thicknesses have a significant effect on pearlite % of CGI. Figure 4a shows sample number 1 (pouring time of 10.53 min and thickness 5 mm) have the lowest value of pearlite % that equal 59.5 and martensite was observed in the microstructure for samples shown in Figure 4a, 4b and 4c which has a thickness of 5, 10 and 15 mm respectively, however, by a further increase in thickness for 20 mm as shown in Figure 4d, pearlite content equals 81.8% and the martensite is shown in very small areas. This implies that the cooling rate attained for the first pouring duration (10.5 min) is high and as result martensite was formed. The results are completely changed by increasing the pouring duration to 17.5 min which shows lower cooling rates for all samples, and the pearlite content increased with a pouring duration of 17.5 min compared with 10.5 min and the martensite is lowered to very small areas as shown in Figure 5.

RETRACTED

**Figure 4:** Pearlite % for sample number 1 with different thicknesses A) Wall thickness 5mm, pearlite % 59.5, B) Wall thickness 10mm, pearlite % 63.60, C) Wall thickness 15mm, pearlite % 62.17, and D) Wall thickness 20mm, pearlite % 81.81.

**Figure 5:** Pearlite % for sample number 2 with different thicknesses: A) Wall thickness 5mm, pearlite % 85.36 and B) Wall thickness 10mm, pearlite % 84.50, C) Wall thickness 15mm, pearlite % 88.89, and D) Wall thickness 20mm, pearlite % 90.11.

### 3.2 Effect of pearlite percentage on Brinell hardness

CGI naturally prefer the synthesis of ferrite matrix rather than pearlite matrix because of the formation of graphite and diffusion of carbon behavior during solidification. Therefore, to enhance a pearlite matrix in CGI pearlite stabilizer elements like that tin and copper must be added to the base iron of GGG70. By comparison between CGI and flake cast iron, the CGI has higher hardness by 10–15% when having the same pearlite content. Engine blocks that manufactured by using completely pearlite matrix have Brinell hardness 179–223, otherwise, cylinder blocks that manufactured by completely pearlite CGI have Brinell hardness between 192-255 vermicular graphite cast iron cylinder blocks containing approximately 70% pearlite has a similar hardness to completely pearlitic grey iron blocks [13]. As shown in Figure 6, the value of hardness for vermicular graphite cast iron reduces with increasing pearlite percent that may be as result of the decrease of martensite formation by decreasing the cooling rates either by longer pouring duration or by increasing the section thickness. The alloying elements increase the tendency to martensite formation by shifting the C-curve to the right-hand side as mentioned before.

**Figure 6:** Pearlite% vs. hardness for sample #1 and sample # 2.

In thin thicknesses (5 mm) for sample #1; it was noticed there is a high percentage of martensite. This area fraction of martensite in sample # 1 for wall thickness (5 mm) equals 22%, however, for sample # 2 (20 mm) equals 4% and these results in lower hardness values for large thicknesses.

RETRACTED

It can be denoted that from Figure 6 for sample number 1 at wall thickness equal 5 mm has a higher value of Brinell hardness 315 because this thickness has a higher % of carbides than around 9%. These carbides due to high cooling rates, so that exist in thin wall sections, also dendrites shapes in microstructures were shown. This defect causes is decreasing in mechanical properties.

Lesser mechanical properties, for example, low hardness is as result of an increase in section thicknesses. There is a relationship between mechanical properties and hardness, thereby values for hardness measurements can be used to predict the tensile strength. The relationship between section thickness and hardness was shown in Figure 7.

**Figure 7:** Brinell hardness vs. section thicknesses in mm.

### 3.3 Percentage on ultimate tensile strength

In thin sections of compacted graphite cast iron casting, the cooling rate has a significant effect because the percentage of nodularity increases as the rate of cooling increases as explained in Figure 8 as nodularity percentage increases this lead to a raise in tensile strength as shown in Figure 8, the tensile strength for sample number 1 has 716 MPa and for sample number 2 has 748 MPa.

**Figure 8:** Tensile strength of 80–100% pearlite content as a function of Nodularity.

The tensile strength in grey cast iron may be a constant value at different thicknesses, but in CGI the tendency of nodularity to increase in thin sections is high, which lead to giving high strength in thin sections rather than thick sections, so CGI has a beneficial effect to use in different applications.

### 3.4 Effect of nodularity percentage on Brinell hardness

The effect of the graphite increasing behavior on hardness is declared on Figure 9. At range (80–100%) pearlite percent, the hardness is increased as a nodularity percent increase; Figure 9 shows the hardness for sample 1 around 289, and hardness for sample 2 around 245.5.

**Figure 9:** Brinell hardness of 80–100% pearlite content as a function of nodularity %.

Table 3 illustrate the section thicknesses effect with a spheroidal number, in which sample #1 the spheroidal number at 5 mm thickness has 150 nodules counts that decrease with the increase in section thickness as being observed in sample #1 for 20 mm thickness that has 58 nodules counts, accordingly sample # 2 has the same behavior, as compared with sample # 1 shown in Figure 10.

**Figure 10:** Section thicknesses vs. spheroidal number for the two samples.

## 4 Conclusions

The microstructure and mechanical characteristics of CGI produced using GGG70 as a starting material with 1% Cu and 0.045% Sn addition with Mg modification have been studied and the followings can be concluded:

1 Longer pouring time (17.5 min) results in 90% pearlite formation, however shorter pouring time (10.5 min) shows only 59.5% pearlite for the same section thickness (5 mm) which is as result of the slower cooling rate obtained for longer pouring time and the elimination of the martensite formation.
2 The increase in the section size decreases the cooling rate and has the same effect to the longer pouring time on the pearlite formation; the pearlite content increases by enlarging the section thickness.
3 Nodularity percentage decreased by longer pouring time and by larger section thickness.
4 Hardness decreased with longer pouring duration and by larger section thickness due to the elimination of the martensite phase in the matrix.
5 The content of Cu and Sn must be adjusted in case of small thickness and shorter pouring duration compacted (vermicular) graphite iron to avoid martensite transformation.

RETRACTED

## Declarations

### Author contribution statement

Mahmoud A. Essam Ahmed Y. Shash, Hassan Megahed & Emad El-Kashif: Conceived and designed the experiments; Performed the experiments; Analyzed and interpreted the data; Contributed reagents, materials, analysis tools or data; Wrote the paper.

### Funding statement

This research did not receive any specific grant from funding agencies in the public, commercial, or not-for-profit sectors.

### Data availability statement

Data will be made available on request.

### Declaration of interests statement

The authors declare no conflict of interest.

### Additional information

No additional information is available for this paper.
